# Combination of the NRF2 Inhibitor and Autophagy Inhibitor Significantly Inhibited Tumorigenicity of Castration-Resistant Prostate Cancer

**DOI:** 10.1155/2022/4182401

**Published:** 2022-06-20

**Authors:** Yong Zhang, Zhixiang Xin, Baijun Dong, Wei Xue

**Affiliations:** Department of Urology, Ren Ji Hospital, School of Medicine, Shanghai Jiao Tong University, Shanghai 200127, China

## Abstract

Prostate cancer (PCa) is the most frequent cancer in men. Developing new treatment methods for CRPC will be a significant challenge in the clinical treatment of PCa. In conclusion, the results of this study show that NRF2 is downregulated in untreated PCa samples compared to normal PCa samples; however, it was upregulated in mCRPC samples compared to HSPC samples. These results demonstrated that NRF2 may serve as a tumor suppressor in tumorigenesis but promote PCa androgen-independent transferring after ADT treatment. Bioinformatics analysis showed that NRF2 was related to multiple signaling, such as the AGE-RAGE pathway, MAPK pathway, NF-kappa B signaling, PI3K-Akt signaling pathway, and VEGF signaling pathway. Moreover, we revealed that the NRF2 inhibitor significantly inhibited tumorigenicity of CRPC cells in vitro. Of note, combination of the NRF2 inhibitor and autophagy inhibitor had a more significantly suppressive role than either ML385 or CQ, indicating that combination of CQ (autophagy inhibitor) and ML385 (NRF2 inhibitor) is a potential treatment of CRPC. Finally, we conformed that high levels of autophagy regulators LC3B, ULK1, and beclin1 significantly correlated to longer PSA recurrence-free survival time. We think that this study could provide more evidence to confirm that NRF2 is a crucial regulator and targeting NRF2 and autophagy is a potential therapy option for CRPC.

## 1. Introduction

Prostate cancer (PCa) is the most frequent cancer in men in Western countries [1]. With the increasing popularity of PCa screening in East Asia, particularly China, the incidence of PCa is rising year by year [2]. The number of patients diagnosed with PCa is rising, and it will soon pose a major threat to global public health. For men with PCa, androgen deprivation therapy (ADT) is the mainstay of treatment. However, most PCas become resistant to ADT after prolonged treatment and progress to castration-resistant PCa (CRPC) [3, 4]. The progression of CRPC is also dependent on androgen receptor- (AR-) related signaling pathways. As a result, a second generation of ADT therapy for AR was created. Unfortunately, after second-generation ADT therapy, almost all CRPC patients progress to AR-independent PCa (AIPC), including small cell carcinoma of the prostate (SCC) and double-negative PCa (DNPC) [5–7]. As a result, developing new treatment methods for CRPC will be a significant challenge in the clinical treatment of PCa.

As a bZIP transcription factor, NRF2, along with small Maf proteins, regulates gene expression via antioxidant response elements (AREs) [8]. ARE is a promoter and enhancer element that responds to ROS, carcinogens, antibiotics, and xenobiotics and regulates basal transcription and antioxidant enzyme induction [9]. Keap1 is a NRF2 binding protein found in the cytoplasm that acts as a negative regulator of NRF2 in vivo. Keap1's ubiquitination, phosphorylation, and nuclear shuttling mechanisms can all influence NRF2 activity [10, 11]. Some studies have found that NRF2 and AR can regulate each other in the prostate, and it is speculated that they, along with AR, may play a critical regulatory role in the formation, development, and treatment of prostate tumors [12, 13]. The crosstalk between AR and NRF2 signaling had been demonstrated in multiple studies [11, 12]. NRF2, for example, has been demonstrated to reduce AR transactivation by increasing nuclear accumulation of p120-NRF1 [11]. Overexpression of NRF2 was demonstrated to dramatically decrease AR activity generated by dihydrotestosterone (DHT) [11]. As a result, targeted NRF2 inhibition is expected to become a new therapeutic modality for the treatment of PCa, particularly in CRPC patients. A large number of clinical trials on autophagy and tumor therapy, on the other hand, are currently underway, but the results are unsatisfactory. It is hypothesized that when autophagy is inhibited, other pathways may take its place. When autophagy is inhibited, cancer cells can rely on NRF2 signaling to maintain protein levels, according to Andrew Thorburn's research team. Therefore, we propose that combination of CQ (autophagy inhibitor) and ML385 (NRF2 inhibitor) is a potential treatment of CRPC.

The current study explored the correlation between NRF2 expression and clinicopathological information of PCa. In addition, the current research investigated the effect of the NRF2 inhibitor in the growth of CRPC cells. We think that this study could provide more evidence to confirm that NRF2 is a crucial regulator and a potential therapy target of CRPC.

## 2. Materials and Methods

### 2.1. Clinical PCa Samples

This study included 472 male patients with PCa who underwent resection or biopsy at Renji Hospital between June 2010 and August 2015. All patients enrolled in this study gave written informed consent to the use of their tissue samples for clinical research purposes. Patients receiving NCHT prior to radical prostatectomy were treated with docetaxel together with goserelin plus bicalutamide. In this study, biochemical recurrence (BCR) was defined as a PSA value of 0.2 ng/ml after RP, confirmed by at least two consecutive measurements.

### 2.2. Enrichment Analysis

The DEGs between NRF2-high PCa and NRF2-low PCa samples were identified by using the “edgeR” R package [14] with a *P* value < 0.01 and ∣logFC | >1. Next, KEGG enrichment analysis was carried out with the DAVID system (https://david.ncifcrf.gov/summary.jsp) [15].

### 2.3. Cell Culture

Human PCa cell lines, including 22Rv1 and DU145, were obtained from the Chinese Academy of Sciences' typical culture collection center (Shanghai, China) and cultured in RPMI-1640 medium supplemented with 10% fetal bovine serum in a 5% CO_2_ atmosphere at 37° C. All regents were purchased from GIBCO (GIBCO; Thermo Fisher Scientific Inc.)

### 2.4. Cell Viability Analysis

CellTiter-Glo 3D cell viability assay was conducted to determine cell viability. Cells were plated in a low-attachment 96-well plate at a density of 200 per well with prostate organoid medium with 2% Matrigel. At the third day of plating, treatments were started by addition of medium containing 10 *μ*M chloroquine (CQ) (Sigma), together with 5 *μ*M ML385 in five technical replicates per treatment group. Following four days of treatment, cell viability of the treated tumor cells was assessed using the CellTiter Glo 3D Reagent (Promega) according to the manufacturer's instructions.

### 2.5. Immunohistochemistry

Immunostaining was performed as previously reported [16]. The proportion of positive cells was calculated in the total number of cells in each field. Areas with strong dyeing intensity are marked as “3,” those with medium intensity are marked as “2,” and those with low and negative intensity are marked as “1 and 0.”

### 2.6. Statistical Analysis

For statistical analysis, GraphPad prism 9 (GraphPad software, USA) was used. We used the *t*-test and Tukey's multiple comparison test to assess the differences between experimental variables. The difference is considered as significant when the *P* value is equal to or less than 0.05.

## 3. Results

### 3.1. TCGA Analysis Showed That NRF2 Was Downregulated in Untreated PCa

In order to evaluate the expression levels of NRF2 in PCa, we firstly analyzed TCGA database. The results showed that NRF2 was downregulated in N0 stage and N1 stage PCa samples compared to the normal sample (Figure 1(a)). However, no significant difference of NRF2 expression between N0 and N1 PCa was observed (Figure 1(a)). Moreover, we found that NRF2 was suppressed in stage 1, stage 2, and stage 3 PCa samples compared to normal samples, however, not significantly differently expressed among different stages of PCa (Figure 1(b)).

### 3.2. NRF2 Protein Levels Was Downregulated in Untreated PCa

Next, we evaluate the protein levels of NRF2 in PCa using human protein atlas database. As present in Figure 1, NRF2 protein levels were significantly lower in high-grade PCa samples compared to low-grade PCa samples (Figure 1(c)).

### 3.3. TCGA Analysis Showed that NRF2 Low Expression Was Correlated to Poor Outcome in Untreated PCa

Then, the PCa samples were divided into NRF2-high and low groups. As present in Figure 2, we observed that the number of death cases was significantly lower in NRF2-high groups (Figure 2(a)). High NRF2 expression levels were found to be substantially linked with a favorable survival rate; however, reduced NRF2 expression was linked to a worse survival rate in PCa (Figure 2(b)).

### 3.4. NRF2 Is Suppressed in Untreated PCa Tissues and Is Associated with Disease Progression

To validate the TCGA dataset, we performed immunohistochemical staining assay by using a tissue chip containing 281 hormone-sensitive PCa specimens established by the department of urology, Renji Hospital. By analyzing the correlation between NRF2 protein levels and clinical data of PCa patients, we revealed higher total, nuclear, and cytoplasm protein levels of NRF2 correlated to longer biochemical recurrence-free (BCR-free) survival time and lower protein levels of NRF2 correlated to shorter BCR-free survival time, which was consistent with TCGA data analysis (Figures 3(a)–3(d)). Finally, we analyzed the Tayler dataset and observed a similar result (Figure 3(e)). Collectively, these results indicated that NRF2 low expression was correlated to poor outcome in PCa.

### 3.5. NRF2 Is Upregulated in mCRPC Samples Compared to HSPC Samples

Next, we detected the protein levels of NRF2 between HSPC and mCRPC samples collecting from the same patient using immunohistochemical staining. Very interestingly, we found that NRF2 was highly expressed in mCRPC samples compared to HSPC samples, indicating that NRF2 was activated during PCa androgen-independent transformation (Figure 4(a)). To further confirm these findings, we detected NRF2 protein levels in HSPC and mCRPC samples using a TMA containing 84 neoadjuvant endocrine therapy (NHT) PCa samples, 54 neoadjuvant endocrine + neoadjuvant chemotherapy (NCHT) PCa samples, 281 untreated PCa samples, and 43 CRPC and 10 SCC samples. The results showed that NRF2 levels were higher in 43 CRPC and 10 SCC samples compared to untreated PCa samples. Interestingly, NRF2 levels were significantly suppressed after neoadjuvant endocrine therapy and lower in 84 neoadjuvant endocrine therapy (NHT) PCa samples and 54 neoadjuvant endocrine + neoadjuvant chemotherapy (NCHT) PCa samples compared to 281 untreated PCa samples (Figure 4(b)). These results indicated that NRF2 protein may have a crucial regulatory role in PCa androgen-independent transformation.

### 3.6. Bioinformatics Analysis of NRF2 in Prostate Cancer

In order to evaluate the mechanism of NRF2 in PCa, we divided all PCa samples into NRF2-high and NRF2-low groups based on the median levels of NRF2. Then, the differently expressed gene between NRF2-high and low groups was identified. As present in Figure 5, a total of 4317 overexpressed genes and 477 suppressed genes were identified in NRF2-high groups (Figure 6(a)). Among them, NFE2L2, LONRF3, OSMR, RAP1B, and PLEKHA1 were the most significantly upregulated genes and SUMF1, FBXO25, INPP5K, IGHMBP2, and BLOC1S3 were the most significantly downregulated genes. Bioinformatics analysis showed that these upregulated DEGs were significantly related to the AGE-RAGE pathway, chemokine signaling, ECM-receptor interaction, focal adhesion, Hippo signaling, leishmaniasis, MAPK pathway, NF-kappa B signaling, PI3K-Akt signaling pathway, Rap1 pathway, TNF pathway, and Th17 cell differentiation (Figure 6(b)). The downregulated DEGs were significantly related to the neurotrophin signaling pathway, neutrophil extracellular trap formation, pyrimidine metabolism, retrograde endocannabinoid signaling, ribosome, systemic lupus erythematosus, thermogenesis, and VEGF signaling pathway (Figure 6(c)).

### 3.7. NRF2 Inhibitor Significantly Inhibited Tumorigenicity of CRPC Cells In Vitro

We used a nonadherent sphere assay to detect whether NRF2 affected the tumorigenic ability of CRPC cells. In 3D cultures, the effects of NRF2 inhibition (ML385) on 22Rv1 and DU145 cell growth were further investigated (Figures 5(a) and 5(c)).

Compared to the control, ML385 significantly suppressed the tumorigenicity of CRPC cells in vitro. The cell viability of DU145 and 22Rv1 cells was suppressed by 79.3% and 44.5%, respectively. The number of DU145 and 22Rv1 cell spheres was decreased by 36.3% and 38.6%, respectively. The Feret diameter of DU145 and 22Rv1 cell spheres was decreased by 41.3% and 23.5%, respectively. Together, these results indicate that ML385 reduced the tumorigenicity of CRPC cells (Figures 5(a)–5(d)).

### 3.8. Combination of the NRF2 Inhibitor and Autophagy Inhibitor Significantly Inhibited Tumorigenicity of CRPC Cells

To evaluate whether the combination of the NRF2 inhibitor and autophagy inhibitor could be a potential therapy strategy for CRPC, we treated DU145 and 22Rv1 cells with the NRF2 inhibitor (ML385) and autophagy inhibitor (CQ). As present in Figure 5, the cell viability, sphere number, and organized size of DU145 and 22Rv1 cells were not affected by CQ treatment (Figures 5(a)–5(d)). Meanwhile, the cell viability, sphere number, and organized size of 22Rv1 cells were slightly suppressed after CQ treatment, indicating that treatment with the autophagy inhibitor (CQ) alone did not affect the tumorigenicity of CRPC cells in vitro (Figures 5(a)–5(d)).

As expected, we found that a combination of the NRF2 inhibitor and autophagy inhibitor had a more significantly suppressive role than either ML385 or CQ. The cell viability of DU145 and 22Rv1 cells was suppressed by 93.1% and 76.5%, respectively, after treatment with combination. The number of DU145 and 22Rv1 cell spheres was decreased by 84.5% and 64.5%, respectively, after treatment with combination. The Feret diameter of DU145 and 22Rv1 cell spheres was decreased by 51.3% and 57.5%, respectively, after treatment with combination (Figures 5(a)–5(d)).

### 3.9. The Dysregulation of Autophagy Markers Was Correlated to the Prognosis of PCa

The abovementioned analysis demonstrated that the combination of the NRF2 inhibitor and autophagy inhibitor significantly suppressed PCa growth. Thus, we detected whether autophagy markers, including LC3B, ULK1, and beclin1, were correlated to PCa prognosis. LC3B, ULK1 and Beclin1 are three important regulators in the regulation of autophagy. Here, we detected whether these autophagy markers were correlated to PCa prognosis. Phosphatidylethanolamine (PE) interconjugates with LC3I in the cytoplasm to generate lipidated forms of LC3II that are embedded in the bilayer membrane. This lipid-bound form of LC3 is often used as a marker for autophagosomes. Beclin1 is phosphorylated by ULK1 and can act as an integral scaffold for the PI3K complex, facilitating the localization of autophagic proteins to autophagic vacuoles. Therefore, we selected these three proteins as markers of autophagy. IHC assay was conducted to analyze LC3B, ULK1, and beclin1 protein levels in prostate tissue specimens.  Figure 7 showed the representative staining of LC3B, ULK1, and beclin1 protein in TMAs. As present in Figure 7(b), we observed that high levels of LC3B, ULK1, and beclin1 significantly correlated to longer BCR-free survival time.

## 4. Discussion

NRF2 is the master regulator of a group of cytoprotective genes that protect cells from environmental stressors such as reactive oxygen species (ROS) and electrophiles [17]. In addition to its importance in cell physiology and stress response, new research has revealed that NRF2-regulated pathways are frequently activated and play a significant role in initiating malignant transformation, providing a growth advantage, and modulating cancer metabolism [18]. About 30% of human lung cancers have Keap1 or nfe2l2 mutations, resulting in the stability of nfe2l2 gene product NRF2, which controls the oxidation balance. NRF2 accumulation in lung cancer stabilizes Bach1 by inducing HO1, an enzyme that breaks down heme [19]. C-myc-directed NRF2 drives the malignant progression of head and neck cancer through the activation of glucose-6-phosphate dehydrogenase and transketolase [20]. NRF2 overexpression is linked to enhanced tumor-infiltrating lymphocytes and tumor immunity in ER-positive/HER2-negative breast cancer [20]. NRF2 activation promotes invasive lung cancer and is associated with adverse clinical outcomes. Decoupling of NRF2 expression in nonsmall cell lung cancer promotes the maintenance of the mesenchymal state. However, the roles of NRF2 in PCa remained to be further explored. In this study, we for the first time revealed that NRF2 was downregulated in untreated PCa samples. Moreover, high NRF2 levels were found to be substantially related with a favorable survival rate in untreated PCa patients. In our study, the positive percentage of NRF2 was less than 20% in untreated patients (data not shown), while that was 100% in SCC patients, which indicated that NRF2 could serve as a marker in the diagnosis of SCC. Thus, we believe that NRF2 plays an important role in castration resistance and even neuroendocrine differentiation. In order to validate the TCGA dataset, we performed immunohistochemical staining assay by using collecting samples and revealed higher total, nuclear, and cytoplasm protein levels of NRF2 correlated to longer BCR-free survival time. These results indicated that NRF2 low expression was correlated to poor outcome in untreated PCa.

ADT is the mainstay of treatment for PCa. However, most PCas become resistant to ADT after prolonged treatment and progress to castration-resistant PCa (CRPC). Understanding the mechanisms underlying the androgen-independent transferring is important for CRPC treatment. Previous studies had demonstrated the interaction between NRF2 signaling and AR signaling. Very interestingly, we found that NRF2 was highly expressed in mCRPC samples compared to HSPC samples, which were higher in 43 CRPC and 10 SCC samples compared to untreated PCa samples and were significantly suppressed after neoadjuvant endocrine therapy and lower in 84 neoadjuvant endocrine therapy (NHT) PCa samples. We used a nonadherent sphere experiment to see if NRF2 altered the tumorigenic potential of CRPC cells and found that ML385 decreased the tumorigenicity of CRPC cells.

Programmed cell death (autophagy, apoptosis, and necrotic ptosis) plays a key role in tumor metastasis and drug resistance [21]. Autophagy plays dual roles in PCa progression via promoting and suppressing PCa growth based on different cellular characteristics. For example, beclin1 is deleted in many PCa patients, which is an important autophagy regulator, suggesting that autophagy may be a tumor-suppressive mechanism in the PCa [22]. Autophagy may also serve as a survival mechanism for cells under stress, making it a tumor-promoting mechanism in PCa. A great number of literatures indicates that the inhibition of AR activity, microtubule, and cell signaling stimulates the adaptive response of autophagy in PCa models. Regulating autophagy can improve the therapeutic effect of the abovementioned treatment on PCa. Autophagy induction has been shown to make cells more susceptible to apoptosis stimulation and radiation in androgen-independent PCa cells [23, 24]. Very interestingly, as a key regulator of autophagy, we found that NRF2 is downregulated in untreated PCa samples compared to normal PCa samples; however, it was upregulated in mCRPC samples compared to HSPC samples. These results further indicated that NRF2 may serve different roles in the progression of PCa and was activated during PCa androgen-independent transformation. Despite that no autophagy-targeting drugs were approved for PCa therapy, several preclinical studies indicated the promising progression about the using of autophagy-related drugs in PCa [25–27]. For example, diosgenin has high antitumor activity in prostate cancer via inducing autophagy [26]. Moreover, Eriocalyxin B (EriB), a promising candidate in cancer therapy, induced apoptosis and autophagy in PCa via AKT-MTOR signaling [27]. Here, we also evaluate the effect of the autophagy inhibitor on PCa growth. We found that treatment with the autophagy inhibitor (CQ) alone did not affect the tumorigenicity of CRPC cells in vitro.

In tumors, a functional link between autophagy dysregulation and NRF2 signaling pathways has been discovered. Recent research has shown that the autophagy and NRF2 signaling pathways are inextricably linked via p62, which binds and transports ubiquitinated protein aggregates to autophagosomes [28]. The interaction of p62 and Keap1 increases NRF2 stability and transcriptional activity. In this study, we found that combination of the NRF2 inhibitor and autophagy inhibitor had a more significantly suppressive role than either ML385 or CQ, indicating that combination of CQ (autophagy inhibitor) and ML385 (NRF2 inhibitor) is a potential treatment of CRPC.

In conclusion, the results of this study show that NRF2 is downregulated in untreated PCa samples compared to normal PCa samples; however, it was upregulated in mCRPC samples compared to HSPC samples. These results demonstrated that NRF2 may serve as an tumor suppressor in tumorigenesis but promote PCa androgen-independent transferring after ADT treatment. Moreover, we revealed that the NRF2 inhibitor significantly inhibited tumorigenicity of CRPC cells in vitro. Of note, combination of the NRF2 inhibitor and autophagy inhibitor had a more significantly suppressive role than either ML385 or CQ, indicating that combination of CQ (autophagy inhibitor) and ML385 (NRF2 inhibitor) is a potential treatment of CRPC.

## Figures and Tables

**Figure 1:** NRF2 was downregulated in untreated PCa. (a) The expression levels of NRF2 in normal prostate, N0 stage, and N1 stage PCa samples were analyzed using TCGA database. (b) The expression levels of NRF2 in normal prostate, stage 1, stage 2, and stage 3 PCa samples were analyzed using TCGA database. (c) The protein levels of NRF2 in PCa were analyzed using Human Protein Atlas database.

**Figure 2:** NRF2 low expression was correlated to poor outcome in untreated PCa. (a) The number of death cases was significant lower in NRF2-high groups. (b) Kaplan-Meier analysis of the correlation between NRF2 expression levels and progression-free survival time in patients with PCa.

**Figure 3:** NRF2 is suppressed in untreated PCa tissues and is associated with disease progression. (a) The representative images of IHC 0, 1, 2, and 3 of nuclear and cytoplasmic levels of NRF2 in PCa. (b) Higher total, (c) nuclear, and (d) cytoplasm protein levels of NRF2 correlated to longer BCR-free survival time. (e) Taylor dataset analysis showed that NRF2 low expression was correlated to poor outcome in PCa.

**Figure 4:** NRF2 is upregulated in mCRPC samples compared to HSPC samples. (a) NRF2 was highly expressed in mCRPC samples compared to HSPC samples. (b) The protein levels of NRF2 in a TMA containing 84 neoadjuvant endocrine therapy (NHT) PCa samples, 54 neoadjuvant endocrine + neoadjuvant chemotherapy (NCHT) PCa samples, 281 untreated PCa samples, and 43 CRPC and 10 SCC samples were detected using IHC methods.

**Figure 5:** Combination of the NRF2 inhibitor and autophagy inhibitor significantly inhibited tumorigenicity of PCa cells. (a) The representative images of PCa 22Rv1 spheres after treatment with the NRF2 inhibitor, autophagy inhibitor, and combination. (b) The cell viability, sphere number, and organized size of PCa 22Rv1 spheres after treatment with the NRF2 inhibitor, autophagy inhibitor, and combination. (c) The representative images of PCa DU145 spheres after treatment with the NRF2 inhibitor, autophagy inhibitor, and combination. (d) The cell viability, sphere number, and organized size of PCa DU145 spheres after treatment with the NRF2 inhibitor, autophagy inhibitor, and combination.

**Figure 6:** Bioinformatics analysis of NRF2 in prostate cancer. (a) The differently expressed genes between NRF2-high and NRF2-low groups were identified. (b, c) KEGG analysis of upregulated and downregulated DEGs in PCa.

**Figure 7:** The dysregulation of autophagy markers was correlated to the prognosis of PCa. (a) The representative images of IHC 0, 1, 2, and 3 levels of LC3B, ULK1, and beclin1 in PCa. (b) high levels of LC3B, ULK1, and beclin1 significantly correlated to longer BCR-free survival time.

## Data Availability

All data generated or analyzed during this study are included in this study.
